# A Nested Case-Control Study of the Relationship between Salivary Inflammatory Mediators, Periodontal Parameters, and Preterm Birth in a Chinese Population

**DOI:** 10.1155/2022/8629680

**Published:** 2022-08-18

**Authors:** Min Wu, Chanjuan Ye, Huijun Li, Xiuqiao Yang, Sujun Zhu, Fangming Zhou, Ying Hao, Shaowu Chen, Shaoyun Jiang

**Affiliations:** ^1^Department of Stomatology, The Affiliated Shenzhen Maternity and Child Healthcare Hospital of the South Medical University, Shenzhen 518048, China; ^2^Department of Obstetrics and Gynecology, The Affiliated Shenzhen Maternity and Child Healthcare Hospital of the South Medical University, Shenzhen 518048, China; ^3^Clinical Laboratory, The Affiliated Shenzhen Maternity and Child Healthcare Hospital of the South Medical University, Shenzhen 518048, China; ^4^Stomatological Center, Peking University Shenzhen Hospital, Guangdong Provincial High-Level Clinical Key Specialty, Guangdong Province Engineering Research Center of Oral Disease Diagnosis and Treatment, Shenzhen 518056, China

## Abstract

**Background:**

To explore whether salivary inflammatory mediators and periodontal indices at different gestational stages can be taken as indicators of preterm birth (PTB).

**Methods:**

This nested case-control study enrolled systemically healthy pregnant women at 9 to 36 weeks of gestation. Periodontal indices were measured at the enrollment date, and interleukin-1*β* (IL-1*β*), IL-6, tumor necrosis factor (TNF-*α*), prostaglandin E2 (PGE2), and 8-hydroxy-deoxyguanosine (8-OHdG) in the saliva were determined by enzyme-linked immunosorbent assay (ELISA). The birth outcome was recorded.

**Results:**

PTB occurred in 26 women. A total of 104 matched women with full-term birth (FTB) were used as controls. The PTB women enrolled at 24-28 gestational weeks displayed a significantly greater bleeding index (BI), probing pocket depth (PD), PD ≥ 4 mm sites (%), saliva-TNF-*α*, and saliva-PGE2 (*P* < 0.05). BI and PGE2 in the saliva were found to be positively associated with PTB (OR = 4.79, *P* = 0.048, 95%CI = 1.014 to 22.628; OR = 1.07, *P* = 0.04, 95%CI = 1.004 to 1.135, respectively). The areas under the receiver operating characteristic curve (ROC) of BI and saliva-PGE2 were 0.82 and 0.78, respectively, and that of the combined detection was 0.91, which was larger than either marker alone, although the differences were not significant (*P* > 0.05).

**Conclusions:**

The combination of BI and PGE2 in saliva at 24-28 gestational weeks could be a predictor of PTB in asymptomatic women. However, the results should be further explored with larger sample size.

## 1. Introduction

Preterm birth (PTB), defined as birth between 28 and 36 weeks of gestation, occurs in 5-18% of pregnancies worldwide, is the leading cause of neonatal morbidity and mortality, and is also the second leading cause of death in children under five years of age [1]. Even with recent advances in neonatal care and improvements in prematurity survival, the preterm delivery rate has continued to increase [2]. Efforts to prevent or reduce the prevalence of PTB seem to be largely unsuccessful. Therefore, the early identification of women at risk for developing PTB and the initiation of preventive measures as early as possible are very important [3].

Current strategies to screen women at risk for developing PTB are mainly based on a previous history of spontaneous preterm delivery, transvaginal cervical length, and fetal fibronectin level [4]. The former is impossible to assess for primiparous women [4], and the latter two are uncertain due to controversial results about their predictive accuracy [4, 5]. Currently, although high-quality ultrasound machines along with skilled ultrasound doctors exist, these tests are not recommended for routine use for screening pregnant women without obvious risk factors for spontaneous preterm birth [4–6].

It is known that inflammation and infection at the maternal-fetal interface may play a major role in the etiology of spontaneous preterm births [3]. To date, a range of inflammatory mediators in various biologic fluids, such as cervicovaginal fluid, amniotic fluid, urine, and plasma, have been assessed to develop sensitive and reliable predictors to identify women who are at risk of PTB. However, the predictive value of these biomarkers is limited [7, 8]. Therefore, the exploration of simple, efficacious, and noninvasive screening strategies for PTB is imperative.

Periodontitis is an inflammatory disease in which microbial factors induce a series of host responses, including the production of inflammatory mediators in periodontal tissue [9]. In 1996, Offenbacher et al. reported a possible association between preterm birth and periodontal infection in a case–control study [10]. To date, most epidemiological studies support a positive association between preterm birth and periodontal disease [11]. Although the underlying pathogenic mechanism involved in this relationship is not clear, the most prevalent hypotheses are that periodontal infection causes increased systemic inflammation, leading to pregnancy complications, and that translocation of oral pathogens into the placenta causes intrauterine infection and inflammation, resulting in prematurity [12].

However, clinical intervention trials aimed at determining the effect of periodontal treatment on adverse pregnancy outcomes have produced controversial results [13]. Most of them suggest that periodontal treatment during pregnancy reduces the risk of adverse pregnancy outcomes, while others have failed to demonstrate such a positive effect [13]. This discrepancy is due to the methods used for estimating gestational age, the inclusion criteria of the selected cases, and inconsistent interventions [13]. Currently, the conclusive evidence demonstrating an association between periodontal inflammation in gestation and adverse pregnancy outcomes is limited.

One study conducted by Tarannum et al. estimated the levels of PGE2 in gingival crevicular fluid (GCF) and serum at 28-32 weeks of gestation in twenty-two pregnant patients. However, this study could not demonstrate an association between GCF-PGE2 levels at 28-32 weeks of gestation and preterm low birth weight (PLBW) [8]. Interleukin- (IL-) 1*β*, IL-6, tumor necrosis factor alpha (TNF-*α*), and prostaglandin E2 (PGE2) are considered markers of the progression and severity of periodontitis and are major triggers of preterm labor [14]. Oxidative stress, defined as an imbalance between oxidants and antioxidants, may be associated with PTB and periodontal disease [15, 16]. 8-OHdG is a biomarker used to quantify DNA damage from oxidative stress [17]. Saliva is an easily accessible biological sample. The excellent consistency between saliva and blood tests makes salivary biomarkers worthy diagnostic tools [18]. Therefore, this study examined the associations between salivary inflammatory mediators, including PGE2, IL-1*β*, IL-6, TNF-*α*, and 8-OHdG, as well as periodontal indices measured at different gestational ages and PTB and evaluated which and when these parameters could be used as risk factors for PTB among pregnant Chinese women.

## 2. Materials and Methods

### 2.1. Study Setting

This nested case control study was conducted at the Affiliated Shenzhen Maternity and Child Health care Hospital of South Medical University from January 2017 to May 2018 after being approved by the Research and Ethics Committee of the hospital (No. 201640) in full accordance with the World Medical Association Declaration of Helsinki (version 2013). Participants were recruited at 9 to 36 weeks of gestation. Each woman completed demographic and medical history questionnaires and provided informed consent at enrollment.

### 2.2. Inclusion and Exclusion Criteria

The inclusion criteria were as follows: 20 to 40 years of age, singleton gestation, and a minimum of 20 natural teeth. The exclusion criteria were systemic or topical antimicrobial/anti-inflammatory therapy within the previous 6 months, previous PTB, cigarette smoking, anxiety (excluded by consultation), chronic systemic disease (e.g., diabetes, hypertension, epilepsy, cardiac disease, lung disease, and renal disease), and any known inflammatory pathologies other than PD, such as genitourinary diseases, a positive test for human immunodeficiency virus (HIV), and multifetal gestation [19]. Gestational age was assessed by ultrasonic examination and the last menstrual date. After a periodontal examination and the collection of saliva, the subjects were instructed on the methods of oral hygiene, including the correct use of a toothbrush, dental floss, or interdental brushes. At delivery, the birth outcomes were recorded. PTB was diagnosed as delivering between the 28th and 36th gestational weeks, including premature rupture of the membranes, spontaneous preterm labor, or both. Full-term birth (FTB) was diagnosed as delivering at ≥37 weeks of gestation without a complicated pregnancy.

### 2.3. Sample Size Calculation

Sample size was defined based on the following assumptions: the prevalence of periodontal disease was approximately 25% in pregnant women and approximately 50% in the PTB population [20–22]. Given a test power of 80%, an alpha of 5%, and a dropout rate of 20%, the sample size was calculated by the following formula:

(1) $$\begin{array}{c} \bar{p}=\frac{\left(p_{0}+Cp_{1}\right)}{\left(1+C\right)},\\ n={\left\{\frac{u_{\alpha }\sqrt{\left(1+\left(1/C\right)\right)\bar{p}\bar{q}}+u_{\beta }\sqrt{p_{0}q_{0}+p_{1}q_{1}/C}}{p_{0}-p_{1}}\right\}}^{2}. \end{array}$$

*C* = 4, p0 is the prevalence of periodontitis in the PTB population (50%), p1 is the prevalence of periodontitis in pregnant women (25%),*α* = 5%, 1-*β*is the test power (80%), and*n*is the minimum number of subjects to be recruited in the PTB group (34). The prevalence of PTB was reported to be 11.38% in Shenzhen in 2015. Given a dropout rate of 20%, the sample size of the cohort should be at least 359.

### 2.4. Periodontal Index Measurements

Full-mouth periodontal examinations were performed by three trained periodontists (M-W, CJ-Y, and HJ-L) using a manual periodontal probe (No. 002-0913, Kangqiao, Shanghai, China). High interexaminer reliability was achieved with a 0.87 kappa test value in the bleeding index and 0.885 intraclass correlation efficient value in the probing pocket depth. The following clinical parameters were assessed at six sites (mesiobuccal, midbuccal, distobuccal, mesiolingual, midlingual, and distolingual) of each tooth, excluding the wisdom teeth: bleeding index (BI): “0” = normal appearing, healthy gingiva, “1” = color changes related to inflammation but no bleeding, “2” = slight bleeding that remains at the point of sampling, “3” = bleeding extending from the point of sampling and flowing around the gingival margin, “4” = profuse bleeding that overflows the gingival margin, and “5” = spontaneous bleeding; probing pocket depth (PD): defined as the distance from the free gingival margin to the bottom of the sulcus [23].

### 2.5. Saliva Sampling

Before the clinical measurements and after gargling with water, 4 to 6 ml of unstimulated saliva sample was collected into a sterile wide-mouth plastic container. The saliva was stored in aliquots at −80°C until analysis.

### 2.6. Enzyme-Linked Immunosorbent Assay (ELISA)

Saliva samples were stored for 60 min at 4°C and then centrifuged at 10,000 × g for 10 min [24]. The supernatants were collected and used to measure IL-1*β*, IL-6, TNF-a, PGE2, and 8-OHDG levels using commercial ELISA kits (R&D Systems Minneapolis, MN, USA) according to the manufacturer's instructions.

### 2.7. Statistical Analyses

Statistical analysis was performed by using SPSS 20.0 (SPSS Statistics, IBM Corporation, New York, USA). The Shapiro–Wilk test was used to determine the normal distribution of the quantitative data. The BI and PD ≥ 4 mm rates were not normally distributed, and nonparametric tests were used. Data are expressed as the median (quartile). The Mann–Whitney *U* test was used for comparisons between PTB and FTB. Maternal saliva levels of PGE2, IL-1*β*, IL-6, TNF-*α*, 8-OHdG, and PD were normally distributed; therefore, parametric tests were used, and the data are expressed as the mean ± standard deviation (SD). A two-sample *t*-test was used for comparisons between two groups. Comparisons between proportions were performed with the chi-square or Fisher's exact test. Logistic regression analysis was used to evaluate whether maternal periodontal parameters and salivary levels of inflammatory mediators were significantly associated with PTB. Finally, the evaluation of the predictive value of parameters for PTB was performed by calculating the area under the receiver operating characteristic (ROC) curve. The optimal cutoff points to estimate Youden's index were selected for the highest sensitivity and specificity. *P* values < 0.05 were considered statistically significant.

## 3. Results

### 3.1. Patient Characteristics

During the study period, a total of 405 systemically healthy pregnant women aged between 20 and 40 years at gestational weeks 9 to 36 were enrolled, of whom 67 dropped out for various reasons: 28 women were lost during follow-up, 2 because of stillbirth, 28 because of pregnancy complications, and 9 because of a lack of saliva data. Finally, 338 subjects were included in the study, as presented in Figure 1.

Twenty-six pregnant women developed PTB (7.69%), and 312 pregnant women experienced FTB (92.31%). The baseline demographic characteristics of the study population are shown in Table 1. There were no statistically significant differences in age, enrolled gestational week, body mass index (BMI), parity history, education levels, ethnicity, health insurance, drinking, brushing time, floss use, or gingival bleeding parameters before pregnancy and during pregnancy between PTB and FTB (*P* > 0.05). Additionally, there were statistically significant differences in the percentage of employed and brushing times, which were lower in the PTB group (*P* < 0.01).

### 3.2. Comparison of Salivary Mediators and Periodontal Indices between the FTB and PTB Groups at Different Gestational Ages

Pregnant women at enrollment were divided into four groups: 9-12 weeks of gestation (A), 13-23 weeks of gestation (B), 24-28 weeks of gestation (C), and 29-36 weeks of gestation (D). The number of pregnant women in (B) with PTB was only 8, and they could not be divided into additional subgroups.

The comparison of periodontal parameters and salivary levels of mediators between PTB and FTB at different gestational weeks is presented in Tables 2–4. Group D was excluded because only one PTB occurred. In every group, per PTB case, 4 FTB cases in age-occupation-educational level balance were selected as controls. Periodontal parameters and salivary mediators in Group A and Group B did not show any statistically significant differences between PTB and FTB, as presented in Tables 2 and 3. Among the 61 women in Group C, 10 pregnant women with PTB displayed significantly greater PD (*P* = 0.02), percent of PD over 4 mm (PD ≥ 4 mm) (*P* = 0.04), BI (*P* = 0.001), TNF-*α* levels (*P* = 0.01), and PGE2 levels (*P* = 0.01) than the 40 controls, as presented in Table 4.

### 3.3. Logistic Regression of Four Variables and PTB

Furthermore, the four variables (BI, PD, TNF-*α*, and PGE2) were entered into multiple logistic regression. BI and PGE2 were found to be significantly associated with PTB (OR = 4.79, *P* = 0.048, 95% CI: 1.014-22.628; OR = 1.07, *P* = 0.04, 95% CI 1.004-1.135, respectively; the former is too wide in 95% CI due to the great variability of the sample), whereas no significant association was found between PD, TNF-*α*, and PTB (*P* < 0.05), as presented in Table 5.

### 3.4. Analysis of the Diagnostic Value of BI and PGE2 in Saliva

The receiver operating characteristic curve (ROC) explored the diagnostic value of BI and PGE2 in saliva, individually and combined, at 24-28 weeks of gestation for predicting PTB, as presented in Table 6 and Figure 2. The area under the ROC (AUC) of BI was 0.82 (95% CI, 0.692-0.943), with a sensitivity of 90.0%, a specificity of 62.5%, and an accuracy of 68.0% for the prediction of PTB. The cutoff point of BI was 1.66. The AUC of PGE2 in saliva was 0.78 (95% CI, 0.630-0.920), with a sensitivity of 90.0%, a specificity of 60.0%, and an accuracy of 66.0% for the prediction of PTB. The cutoff point of PGE2 in saliva was 117.70 pg/ml. Combining BI with PGE2 in saliva resulted in an AUC of 0.91 (95% CI, 0.805-1.000), with a sensitivity of 90.0%, a specificity of 87.5%, and an accuracy of 88.0% for the prediction of PTB. Compared with BI and saliva-PGE2 alone, the specificity and accuracy of the combined detection increased for predicting PTB and were larger than either individual marker, although the differences were not significant (*P* > 0.05). The cutoff points of the two indices were 1.25 and 109.75 pg/ml.

## 4. Discussion

This nested case-control study provided some evidence for the association between salivary inflammatory mediators as well as periodontal indices and PTB and possibly predictive parameters of PTB at specific stages in pregnant women without a previous history of spontaneous preterm delivery. To our knowledge, this is the first time to explore in which stage during pregnancy these periodontitis-related parameters could be used as risk factors for PTB.

In the present study, many known risk factors for PTB, such as a previous history of PTB, anxiety, multiple pregnancy, pregnancy complications, and cigarette smoking, were excluded. Meanwhile, among the demographic characteristics and baseline risk factors between PTB and FTB, there were only statistically significant differences in the percentage of employment and brushing times, which were lower in the PTB group. Whether the unemployment existed only during the pregnant period could not be confirmed; thus, the influence of occupation on PTB needs to be further explored.

To exclude the effects of sex hormones on the periodontitis-related parameters as much as possible and search for the exact time point of these parameter differences, grouping of all of the recruited pregnant women was conducted based on the gestational age.

The salivary levels of 8-OHdG, IL-1*β*, and IL-6 were measured in the present study and showed no significant differences between PTB and FTB in every group. Although 8-OHdG in saliva increased during pregnancy [25], serum IL-6 in the third trimester of pregnancy was higher than in the first trimester [26], which did not provide any information about the difference between PTB and FTB. In our previous study [19], IL-1*β*in GCF did not change during pregnancy. Prostaglandins (PGs) are considered one of the key mediators of preterm labor. The concentration of biologically active PGE2 in the amniotic fluid is significantly higher in women with preterm labor [27]. IL-1*β*, IL-6, and TNF-*α* have been suggested to directly stimulate PGE2 production from amnion cells, and this may indirectly initiate premature labor [28]. In this study, TNF-*α* increased in the PTB group, which might enhance PGE2 salivary levels. PGE2 also has many proinflammatory effects on periodontal tissues [8]. Early in 1998, a case-control study suggested that the mothers of PLBW infants had a higher mean GCF-PGE2 level than the mothers of normal birth weight (NBW) infants [29]. However, this case-control study did not report it had any predictive value. In a cohort study, pregnant women with moderate periodontitis and strict plaque control at 28-32 weeks of gestation were recruited, in which GCF-PGE2 levels could not be shown to be a predictor for PLBW [8]. These results are not consistent with ours. This discrepancy may be due to the differences in sample source (i.e., saliva vs. GCF), timing of the sampling (i.e., 24-28 weeks of gestation vs. 28-32 weeks of gestation), and periodontal disease status of the enrolled subjects. Ghallab found that the elements in saliva reflected the activity of whole mouth inflammatory status [9] and were not similar to GCF. Regarding periodontal disease status, Tarannum et al. enrolled pregnant women with moderate periodontitis (≥3 mm attachment loss at no more than 30% of sites), which is different from our study [8].

Periodontal indices included plaque index (PLI), PD, BI, and clinical attachment loss (CAL); however, only PD and BI were detected in this study. CAL was not measured because CAL is the accumulated result of periodontal history and does not reflect the current situation. Meanwhile, the reasons for excluding PLI and CAL from the present study were as follows. First, the periodontal indices except PLI and CAL increase significantly throughout pregnancy after oral hygiene instruction according to our previous study and other studies [19, 30, 31]. Second, it was imperative to limit the examination time and potential discomfort to a minimum to ensure the sufficient recruitment of pregnant women [15, 32]. The status of BI, as an indicator of clinical periodontal conditions, might be a more sensitive index for pregnant subjects, but it may be affected by hormonal changes during pregnancy [19]. One prospective study with 19 pregnant women found a decrease in bleeding on probing scores from 41.2% at 12 weeks of pregnancy to 26.6% at 4-6 weeks postpartum without interventions, while no significant differences in PD and PD > 4 mm between 12 weeks of pregnancy and postpartum were found [33]. In this study, BI, except PD, was associated with PTB after logistic regression, even though PD was different between PTB and FTB in women at 24-28 weeks of gestation.

In the present study, there was no obvious correlation between the periodontal indices and inflammatory mediators at the saliva level (data not shown). These results are consistent with our previous study in which sex hormones enhanced gingival inflammation without affecting inflammatory mediators [19]. Although, in other research, salivary inflammatory mediators were associated with periodontal indices, in addition to the effects of hormones during pregnancy [8], these differences may be due to the severity of periodontal inflammation recruited in these studies [9].

We measured inflammatory mediators in saliva samples from different time points to find the exact time point to show differences between PTB and FTB. Some studies have demonstrated that 24-28 weeks of gestation may be a sensitive period for monitoring the possibility of PTB [5, 34]. Our study showed that the periodontal indices and biomarkers in saliva at 9-12 and 13-23 weeks of gestation revealed no statistically significant differences between PTB and FTB. However, periodontal index BI and salivary PGE2 at 24-28 weeks of gestation could predict the occurrence of PTB. BI and PGE2 were found to be significantly associated with PTB (OR = 4.79, *P* = 0.048, 95% CI: 1.014-22.628; OR = 1.07, *P* = 0.04, 95% CI: 1.004-1.135, respectively; the former is wide in 95% CI due to the great variability of the sample). The results from the logistic regression showed that for each unit increase in BI, the risk of preterm birth increased 4.79 times and, for each 1 pg/ml increase in salivary PGE2, the risk of preterm birth increased by 1.07 times. Meanwhile, the combination of BI and salivary PGE2 was the best indicator, in which the cutoff points of the two indices were 1.25 and 109.75 pg/ml. This time point for predicting the occurrence of PTB is consistent with other studies [5, 34].

Some important study limitations should be pointed out, while interpreting the results of the present study, such as the small samples in the subgroups and the small number of positive events. Based on the prevalence of PTB which was reported in Shenzhen in 2015 at 11.38%, the number of positive events was too small, which may have an impact on the results. Nevertheless, very rigid exclusion criteria were applied when selecting the subjects, and meantime, very rigid age-occupation-educational level balance was used to select controls, in order to eliminate all the other confounding factors as possible. Thus, this study provides possible references for predicting PTB.

In summary, within the limitations of this study, elevated maternal BI and PGE2 salivary levels at 24-28 weeks of gestation may be predictive of PTB. A combination of maternal BI and PGE2 salivary levels at 24-28 weeks of gestation could serve as predictive markers of PTB in women without a previous history of spontaneous preterm delivery. Further studies with a larger sample size are needed to explore these findings.

## Figures and Tables

**Figure 1:** Flow chart of the study.

**Figure 2:** ROC curve of alone and combined detection of BI and saliva-PGE2 levels.

**Table 1:** Demographic characteristics at enrollment in FTB and PTB group.

Demographic variable	FTB (*n* = 312)	PTB (*n* = 26)	*P* value
Mean age (years)	30.41 ± 3.88	31.73 ± 4.17	0.10
Gestation weeks (weeks)	19.29 ± 7.37	19.15 ± 7.49	0.93
BMI (kg/m^2^)	22.05 ± 2.96	21.64 ± 2.85	0.53
Prior deliveries	94 (30.1%)	8 (32.0%)	0.85
Occupation	266 (85.3%)	13 (50.0%)	<0.01^∗^
Education			0.72
≤High school	53 (17.0%)	3 (11.5%)	
≥College	259 (83.0%)	23 (88.5%)	
Ethnicity			0.43
Han	304 (97.4%)	26 (100%)	
Minority	8 (2.6%)	0 (0%)	
Health insurance	307 (98.4%)	26 (100%)	1.00
Alcohol	16 (5.2%)	3 (11.5%)	0.16
Brushing times			0.02^∗^
Once a day	20 (6.4%)	5 (19.2%)	
Twice a day or more	292 (93.6%)	21 (80.8%)	
Brushing time			1.00
No more than 3 minutes	279 (89.4%)	23 (88.5%)	
More than 3 minutes	33 (10.6%)	3 (11.5%)	
Dental floss	89 (28.5%)	7 (26.9%)	0.96
Supragingival scaling history	147 (47.1%)	12 (46.2%)	0.88
Bleeding gum before pregnancy	167 (53.5%)	11 (42.3%)	0.37
Bleeding gum during pregnancy	177 (56.7%)	15 (57.7%)	0.76

^∗^ *P* < 0.05. FTB: full term birth; PTB: preterm birth.

**Table 2:** Periodontal indexes and PGE2, IL-1*β*, IL-6, TNF-*α*, and 8-OHdG salivary levels in PTB and FTB in group A.

Variables	FTB control (*n* = 79)	Nested control (*n* = 28)	PTB (*n* = 7)	*P* value (FTB control)	*P* value (nested control)
PD (mm)	2.61 ± 0.63	2.75 ± 0.64	2.21 ± 0.66	0.12	0.054
PD ≥ 4 mm (%)	5.36 (1.04 to 15.78)	5.36 (0.60 to 19.64)	3.93 (0 to 8.19)	0.21	0.35
BI	2.00 (1.43 to 2.61)	2.03 (1.29 to 2.61)	1.90 (1.06 to 2.46)	0.16	0.29
TNF-*α* (pg/ml)	13.67 ± 2.64	14.05 ± 2.47	14.47 ± 2.03	0.27	0.68
IL-1*β* (pg/ml)	13.37 ± 2.31	13.84 ± 1.87	13.98 ± 1.47	0.49	0.86
PGE2 (pg/ml)	110.02 ± 18.80	111.15 ± 18.48	119.47 ± 20.19	0.21	0.30
IL-6 (pg/ml)	3.28 ± 0.64	3.28 ± 0.69	3.51 ± 0.84	0.38	0.45
8-OHdG (pg/ml)	53.81 ± 14.92	58.13 ± 15.99	53.43 ± 17.17	0.32	0.50

^∗^ *P* < 0.05;  ^∗∗^*P* < 0.01. BI: bleeding index; FTB: full term birth; PTB: preterm birth; IL-1*β*: interleukin-1*β*; IL-6: interleukin-6; 8-OHdG: 8-hydroxy-deoxyguanosine; PD: probing depth; PGE2: prostaglandin E2; TNF-*α*: tumor necrosis factor-*α*.

**Table 3:** Periodontal indexes and PGE2, IL-1*β*, IL-6, TNF-*α*, and 8-OHdG salivary levels in PTB and FTB in group B.

Variables	FTB control (*n* = 133)	Nested control (*n* = 32)	PTB (*n* = 8)	*P* value (FTB control)	*P* value (nested control)
PD (mm)	2.56 ± 0.66	2.47 ± 0.61	2.55 ± 0.75	0.98	0.76
PD ≥ 4 mm (%)	5.66 (0.67 to 16.07)	4.49 (0.94 to 10.21)	11.31 (3.21 to 17.26)	0.47	0.28
BI	1.95 (1.42 to 2.68)	1.83 (1.51 to 2.56)	1.77 (1.38 to 2.64)	0.83	0.86
TNF-*α* (pg/ml)	13.36 ± 2.85	12.99 ± 2.91	12.49 ± 1.88	0.40	0.64
IL-1*β* (pg/ml)	14.03 ± 2.54	14.07 ± 2.38	13.81 ± 2.79	0.81	0.78
PGE2 (pg/ml)	108.75 ± 22.72	109.99 ± 21.70	111.17 ± 26.16	0.77	0.90
IL-6 (pg/ml)	3.20 ± 0.86	3.10 ± 0.92	2.87 ± 0.71	0.28	0.51
8-OHdG (pg/ml)	57.18 ± 15.65	54.51 ± 11.09	55.99 ± 18.44	0.84	0.77

^∗^ *P* < 0.05;  ^∗∗^*P* < 0.01. BI: bleeding index; FTB: full term birth; PTB: preterm birth; IL-1*β*: interleukin-1*β*; IL-6: interleukin-6; 8-OHdG: 8-hydroxy-deoxyguanosine; PD: probing depth; PGE2: prostaglandin E2; TNF-*α*: tumor necrosis factor-*α*.

**Table 4:** Periodontal indexes and PGE2, IL-1*β*, IL-6, TNF-*α*, and 8-OHdG salivary levels in PTB and FTB in group C.

Variables	FTB control (*n* = 61)	Nested control (*n* = 40)	PTB (*n* = 10)	*P* value (FTB control)	*P* value (nested control)
PD (mm)	2.46 ± 0.55	2.42 ± 0.44	2.77 ± 0.33	0.09	0.02^∗^
PD ≥ 4 mm (%)	4.17 (1.20 to 14.51)	4.17 (1.51 to 12.80)	13.10 (3.89 to 28.23)	0.09	0.04^∗^
BI	1.58 (1.25 to 2.10)	1.54 (1.24 to 1.91)	2.75 (1.97 to 3.07)	0.004^∗∗^	0.001^∗∗^
TNF-*α* (pg/ml)	13.22 ± 3.04	12.79 ± 2.82	15.47 ± 1.63	0.045^∗^	0.01^∗^
IL-1*β* (pg/ml)	14.64 ± 2.76	14.65 ± 2.70	14.46 ± 2.23	0.86	0.84
PGE2 (pg/ml)	118.80 ± 22.75	111.84 ± 18.65	130.52 ± 14.38	0.03^∗^	0.01^∗^
IL-6 (pg/ml)	3.21 ± 0.94	3.27 ± 0.92	3.62 ± 0.79	0.25	0.27
8-OHdG (pg/ml)	54.23 ± 18.85	53.62 ± 12.77	61.48 ± 12.72	0.30	0.09

^∗^ *P* < 0.05;  ^∗∗^*P* < 0.01. BI: bleeding index; FTB: full term birth; PTB: preterm birth; IL-1*β*: interleukin-1*β*; IL-6: interleukin-6; 8-OHdG: 8-hydroxy-deoxyguanosine; PD: probing depth; PGE2: prostaglandin E2; TNF-*α*: tumor necrosis factor-*α*.

**Table 5:** Logistic regression analysis of variables and PTB.

Variables	Crude OR	Adjust OR	*P* value	95% CI
BI	5.36	4.79	0.048^∗^	1.014 to 22.628
PD	12.65	3.23	0.41	0.202 to 51.547
PGE2 (pg/ml)	1.07	1.07	0.04^∗^	1.004 to 1.135
TNF-*α* (pg/ml)	1.52	1.35	0.16	0.891 to 2.041

BI: bleeding index; CI: confidence interval; OR: odds ratio; PD: probing depth; PGE2: prostaglandin E2; TNF-*α*: tumor necrosis factor-*α*.

**Table 6:** ROC curve of alone and combined detection of BI and saliva-PGE2 levels.

Variables	Cut off point	AUC	Sensitivity	Specificity
BI	1.66	0.82	90.0	62.5
PGE2 (pg/ml)	117.70	0.78	90.0	60.0
BI+PGE2 (pg/ml)	BI: 1.25 PGE2: 109.75	0.91	90.0	87.5

BI: bleeding index; PGE2: prostaglandin E2; AUC: the area under ROC; sensitivity and specificity were percentages.

## Data Availability

The data that support the findings of this study are available from the corresponding author upon reasonable request.

## References

[1] Harrison M. S., Goldenberg R. L. (2016). Global burden of prematurity. *Seminars in Fetal and Neonatal Medicine*.

[2] Sepúlveda-Martínez A., Díaz F., Muñoz H., Valdés E., Parra-Cordero M. (2017). Second-trimester anterior cervical angle in a low-risk population as a marker for spontaneous preterm delivery. *Fetal Diagnosis and Therapy*.

[3] Wei S. Q., Fraser W., Luo Z. C. (2010). Inflammatory cytokines and spontaneous preterm birth in asymptomatic women: a systematic review. *Obstetrics and Gynecology*.

[4] Esplin M. S., Elovitz M. A., Iams J. D. (2017). Predictive accuracy of serial transvaginal cervical lengths and quantitative vaginal fetal fibronectin levels for spontaneous preterm birth among nulliparous women. *JAMA*.

[5] Abuelghar W. M., Ellaithy M. I., Swidan K. H., Allam I. S., Haggag H. M. (2019). Prediction of spontaneous preterm birth: salivary progesterone assay and transvaginal cervical length assessment after 24 weeks of gestation, another critical window of opportunity. *The Journal of Maternal-Fetal & Neonatal Medicine*.

[6] Rosenbloom J. I., Raghuraman N., Temming L. A. (2020). Predictive value of midtrimester universal cervical length screening based on parity. *Journal of Ultrasound in Medicine*.

[7] Bandoli G., Jelliffe-Pawlowski L. L., Feuer S. K. (2018). Second trimester serum cortisol and preterm birth: an analysis by timing and subtype. *Journal of Perinatology*.

[8] Tarannum F., Faizuddin M., Madaiah H. (2011). Gingival crevicular fluid prostaglandin E2 level as a predictor of preterm low birth weight: a pilot investigation. *Journal of Oral Science*.

[9] Ghallab N. A. (2018). Diagnostic potential and future directions of biomarkers in gingival crevicular fluid and saliva of periodontal diseases: review of the current evidence. *Archives of Oral Biology*.

[10] Offenbacher S., Katz V., Fertik G. (1996). Periodontal infection as a possible risk factor for preterm low birth weight. *Journal of Periodontology*.

[11] Manrique‐Corredor E. J., Orozco‐Beltran D., Lopez‐Pineda A., Quesada J. A., Gil‐Guillen V. F., Carratala‐Munuera C. (2019). Maternal periodontitis and preterm birth: systematic review and meta-analysis. *Community Dentistry and Oral Epidemiology*.

[12] Komine-Aizawa S., Aizawa S., Hayakawa S. (2019). Periodontal diseases and adverse pregnancy outcomes. *Journal of Obstetrics and Gynaecology Research*.

[13] López N. J., Uribe S., Martinez B. (2015). Effect of periodontal treatment on preterm birth rate: a systematic review of meta-analyses. *Periodontology*.

[14] Puertas A., Magan-Fernandez A., Blanc V. (2018). Association of periodontitis with preterm birth and low birth weight: a comprehensive review. *The Journal of Maternal-Fetal & Neonatal Medicine*.

[15] Moore T. A., Ahmad I. M., Zimmerman M. C. (2018). Oxidative stress and preterm birth: an integrative review. *Biological Research for Nursing*.

[16] Chapple J. L. C., Matthews J. B. (2007). The role of reactive oxygen and antioxidant species in periodontal tissue destruction. *Periodontology*.

[17] Yang X., Li C., Pan Y. P. (2016). The influences of periodontal status and periodontal pathogen quantity on salivary 8-hydroxydeoxyguanosine and Interleukin-17 levels. *Journal of Periodontology*.

[18] Eftekhari A., Hasanzadeh M., Sharifi S., Dizaj S. M., Khalilov R., Ahmadian E. (2019). Bioassay of saliva proteins: the best alternative for conventional methods in non-invasive diagnosis of cancer. *International Journal of Biological Macromolecules*.

[19] Wu M., Chen S.-W., Su W.-L. (2016). Sex hormones enhance gingival inflammation without affecting IL-1*β* and TNF-*α* in periodontally healthy women during pregnancy. *Mediators of Inflammation*.

[20] Wu M., Liu S., Chen S. (2007). A case-control study on periodontal status between pre-term and full-term. *Journal of Practical Stomatology*.

[21] Nabet C., Lelong N., Colombier M. L. (2010). Maternal periodontitis and the causes of preterm birth: the case–control Epipap study. *Journal of Clinical Periodontology*.

[22] Santos-Pereira S. A., Giraldo P. C., Saba-Chujfi E. (2007). Chronic periodontitis and pre-term labour in Brazilian pregnant women: an association to be analysed. *Journal of Clinical Periodontology*.

[23] Gürsoy M., Pajukanta R., Sorsa T., Könönen E. (2008). Clinical changes in periodontium during pregnancy and post-partum. *Journal of Clinical Periodontology*.

[24] Sezer U., Ciçek Y., Canakçi C. F. (2012). Increased salivary levels of 8-hydroxydeoxyguanosine may be a marker for disease activity for periodontitis. *Disease Markers*.

[25] Gümüş P., Emingil G., Öztürk V. Ö., Belibasakis G. N., Bostanci N. (2015). Oxidative stress markers in saliva and periodontal disease status: modulation during pregnancy and postpartum. *BMC Infectious Diseases*.

[26] Fu Y. Y., Tang L. L., Hu M., Xiang Z., Hu Y. (2020). Changes of serum interleukin-6 in healthy pregnant women and establishment of relevant reference intervals. *Clinica Chimica Acta*.

[27] Vrachnis N., Karavolos S., Iliodromiti Z. (2012). Review: impact of mediators present in amniotic fluid on preterm labour. *In Vivo*.

[28] Furuta I., Yamada H., Sagawa T., Fujimoto S. (2000). Effects of inflammatory cytokines on prostaglandin E_2_ production from human amnion cells cultured in serum-free condition. *Gynecologic and Obstetric Investigation*.

[29] Offenbacher S., Jared H. L., O'Reilly P. G. (1998). Potential pathogenic mechanisms of periodontitis associated pregnancy complications. *Annals of Periodontology*.

[30] Figuero E., Carrillo-de-Albornoz A., Martín C., Tobías A., Herrera D. (2013). Effect of pregnancy on gingival inflammation in systemically healthy women: a systematic review. *Journal of Clinical Periodontology*.

[31] Patil P., Kashetty M., Kumbhar S., Patil S. (2018). Oral hygiene status, gingival status, periodontal status, and treatment needs among pregnant and nonpregnant women: a comparative study. *Journal of Indian Society of Periodontology*.

[32] Teles R. P., Likhari V., Socransky S. S., Haffajee A. D. (2009). Salivary cytokine levels in subjects with chronic periodontitis and in periodontally healthy individuals: a cross-sectional study. *Journal of Periodontal Research*.

[33] Bieri R. A., Adriaens L., Spörri S., Lang N. P., Persson G. R. (2013). Gingival fluid cytokine expression and subgingival bacterial counts during pregnancy and postpartum: a case series. *Clinical Oral Investigations*.

[34] Zhou Z. J., Bian C. X., Luo Z. W. (2019). Progesterone decreases gut permeability through upregulating occludin expression in primary human gut tissues and Caco-2 cells. *Scientific Reports*.

